This article has been retracted.

# Antibiotics Threaten Wildlife: Circulating Quinolone Residues and Disease in Avian Scavengers

**DOI:** 10.1371/journal.pone.0001444

**Published:** 2008-01-16

**Authors:** Jesús Á. Lemus, Guillermo Blanco, Javier Grande, Bernardo Arroyo, Marino García-Montijano, Felíx Martínez

**Affiliations:** 1 Departamento de Ecología Evolutiva, Museo de Ciencias Naturales, Consejo Superior de Investigaciones Científicas (CSIC), Madrid, Spain; 2 Instituto de Investigación en Recursos Cinegéticos (IREC), Consejo Superior de Investigaciones Científicas (CSIC), Universidad de Castilla-La Mancha (UCLM), Junta de Comunidades de Castilla-La Mancha (JCCM), Ciudad Real, Spain; 3 GIR Diagnostics SL, Madrid, Spain; University of Sydney, Australia

## Abstract

Antibiotic residues that may be present in carcasses of medicated livestock could pass to and greatly reduce scavenger wildlife populations. We surveyed residues of the quinolones enrofloxacin and its metabolite ciprofloxacin and other antibiotics (amoxicillin and oxytetracycline) in nestling griffon *Gyps fulvus*, cinereous *Aegypius monachus* and Egyptian *Neophron percnopterus* vultures in central Spain. We found high concentrations of antibiotics in the plasma of many nestling cinereous (57%) and Egyptian (40%) vultures. Enrofloxacin and ciprofloxacin were also found in liver samples of all dead cinereous vultures. This is the first report of antibiotic residues in wildlife. We also provide evidence of a direct association between antibiotic residues, primarily quinolones, and severe disease due to bacterial and fungal pathogens. Our results indicate that, by damaging the liver and kidney and through the acquisition and proliferation of pathogens associated with the depletion of lymphoid organs, continuous exposure to antibiotics could increase mortality rates, at least in cinereous vultures. If antibiotics ingested with livestock carrion are clearly implicated in the decline of the vultures in central Spain then it should be considered a primary concern for conservation of their populations.

## Introduction

Antibiotics (formally antimicrobials) are one of the biomedical revolutions of the 20^th^ century. Nonetheless, their misuse has led to an increase in diseases in humans and domestic animals worldwide [1]. Huge quantities of antibiotics are used annually in livestock farming operations throughout the world, but the eventual fate of their residues and their potential damage to environmental health generally remains unknown [2], [3].

Withdrawal periods and residue controls are conducted in slaughterhouses to prevent harmful drug residuals in food that humans consume [4]. However, these waiting periods do not apply to carcasses and other wastes disposed of in dumps exploited by scavengers. Therefore, scavengers may consume drug residues in livestock carrion. The use of antibiotics and other drugs in livestock may directly damage the health and survival of scavengers if ingested as toxic residues [5]–[7]. Indirect effects on health may include the acquisition of antibiotic-resistant bacteria [4]–[8] and the alteration of normal protective flora through the acquisition of transient flora that may include pathogenic bacteria [8]–[11]. Furthermore, antibiotic residues ingested by avian scavengers may select for antibiotic resistance, the emergence, dissemination and persistence of which represents a major health problem in human and veterinary medicine worldwide [1], [4].

The “vulture crisis” on the Indian subcontinent caused by diclofenac, of which the use on livestock is banned in the European Union, demonstrates the potential of veterinary drugs to cause massive wildlife mortalities [7]. In Spain, after the bovine spongiform encephalopathy crisis, the ban on abandoning carcasses of free-range livestock in the countryside closed most traditional disposal sites for livestock carcasses used by avian scavengers as food sources [12]. Since then the diet of avian scavengers has been mainly composed of intensively farmed livestock carrion (swine and poultry) treated with antibiotics and other veterinary drugs, which represents the only livestock carrion available for scavengers [8], [9]. Thus, antibiotic residues from treated livestock could pass to scavengers and reduce their populations [8], [12], [13].

We investigated the possible transmission of antibiotic residues from livestock carcasses to nestlings of three vulture species in central Spain (griffon vulture, *Gyps fulvus*, cinereous vulture, *Aegypius monachus* and Egyptian vulture, *Neophron percnopterus*). We also searched for antibiotic residues in liver samples from dead cinereous vultures in the same area, and assessed their potential effects in this and other organs by histopathological analyses. The potential relationships between circulating antibiotic residues and the presence of bacterial and fungal pathogens causing severe disease were also evaluated in the three vulture species. Finally, we assessed whether disease-mediated mortality was associated with the presence of circulating antibiotics in cinereous vultures.

## Results

### Antibiotic residues in livestock carrion

Results of the Four Plate Test of bacterial growth inhibition to detect antibiotic residues (see Material and methods) showed their presence in 21 of 29 samples (72%) from several tissues of swine carcasses available to vultures, varying from 40% of liver to 100% of kidney samples. This suggests that vultures may ingest antibiotics when feeding on livestock carrion.

### Circulating antibiotic residues

We found a high proportion of nestlings carrying circulating antibiotics, especially in Egyptian and cinereous vultures (Table 1). In the three species, enrofloxacin and its metabolite ciprofloxacin showed the highest prevalences and concentrations alone or in combination with other antibiotics (Table 1).

**Table 1:** Antibiotic residues in nestlings of three vulture species in central Spain and their concentrations in plasma.

	Number of samples with antibiotics (%)	Concentration (µg/ml) mean±SD (range)	*n*
Griffon vulture (*n* = 50)			
Antibiotic residues (total)^a^	6 (12)		
Quinolones (total)^b^	6 (12)		
Enrofloxacin	1 (2)	0.16±0.028 (0.14–0.18)	2
Ciprofloxacin	3 (6)	0.077±0.056 (0.025–0.17)	5
Amoxicillin	0 (0)	0.005*	1
Oxytetracycline	0 (0)		
Enrofloxacin+Ciprofloxacin	1 (2)		
Ciprofloxacin+Amoxicillin	1 (2)		
Cinereous vulture (*n* = 49)			
Antibiotic residues (total)^a^	28 (57)		
Quinolones (total)^b^	26 (53)		
Enrofloxacin	7 (14)	0.073±0.076 (0.0005*–0.21)	12
Ciprofloxacin	14 (29)	0.095±0.059 (0.025–0.21)	16
Amoxicillin	2 (4)	0.027±0.037 (0.005*–0.07)	3
Oxytetracycline	0 (0)	0.005±0.000*	2
Enrofloxacin+Ciprofloxacin	2 (4)		
Enrofloxacin+Amoxicillin	1 (2)		
Enrofloxacin+Oxytetracycline	2 (4)		
Egyptian vulture (*n* = 25)			
Antibiotic residues (total)^a^	10 (40)		
Quinolones (total)^b^	6 (24)		
Enrofloxacin	2 (8)	0.104±0.116 (0.0005*–0.28)	5
Ciprofloxacin	0 (0)	0.078±0.026 (0.04–0.10)	4
Amoxicillin	2 (8)	0.061±0.112 (0.005*–0.23)	4
Oxytetracycline	1 (4)	0.005±0.000*	2
Enrofloxacin+Ciprofloxacin	3 (12)		
Ciprofloxacin+Amoxicillin	1 (4)		
Amoxicillin+Oxytetracycline	1 (4)		

* Values corresponding to the half of the detection limit.

a Pooling all different antibiotics.

b Pooling enrofloxacin and ciprofloxacin.

Eight additional fledglings and one adult cinereous vulture from the same colony (as identified by leg rings previously applied) which had not been sampled for blood in their nests, were treated in rehabilitation centres in 2002 and 2005. All had one to three antibiotics in plasma (ciprofloxacin = 67%, enrofloxacin 89%, amoxicillin 11%, oxytetracycline 11%) at high mean concentrations (ciprofloxacin = 0.15±0.066 µg/ml, *n* = 6, enrofloxacin = 0.089±0.049 µg/ml, *n* = 8, amoxicillin = 0.09 µg/ml, *n* = 1, oxytetracycline = 0.005 µg/ml, *n* = 1).

Residues of both enrofloxacin and ciprofloxacin were found in all samples of liver tissue from nine dead cinereous vultures at mean concentrations of 0.18±0.11 µg/g (range 0.08–0.21 µg/g) and 0.09±0.04 µg/g (range 0.03–0.07 µg/g) respectively.

### Relationships between circulating antibiotics, disease and mortality

Variable prevalences of bacterial and fungal pathogens involved in severe disease were found in the sampled nestlings (Table 2). A proportion of cinereous (16.3%, *n* = 49) and Egyptian (4.0%, *n* = 25) vultures were infected with two or more of these pathogens.

**Table 2:** Prevalence (% of infected individuals) of each pathogen in nestlings of three vulture species from central Spain.

	Egyptian vulture *n* = 25	Cinereous vulture *n* = 49	Griffon vulture *n* = 50
*Salmonella* sp	32	16	0
*typhimurium*	50	25	-
*enteritidis*	25	75	-
*gallinarum*	12.5	-	-
*pullorum*	12.5	-	-
*Mycobacterium avium* (serotype 7)	4	8	0
*Candida albicans*	0	26.5	6
*Aspergillus fumigatus*	9	16	0
Total	32	53	6

Prevalence of each *Salmonella* serotype was calculated from the total positive isolates in each vulture species (*n* = 8 for both Egyptian and cinereous vultures).

The presence of antibiotic residues was clearly associated with the presence of pathogens in the three vulture species (Fig. 1). Pathogen prevalence was only related to the presence of quinolones in the vulture species (cinereous and Egyptian) in which there were a sufficient number of samples with several antibiotics (log-linear analyses, both *P*<0.00001, goodness-of-fit, both *P*>0.855).

**Figure 1:** Relationships between prevalence of pathogens (% of individuals with pathogens) and the presence or absence of antibiotics in plasma of nestlings of three vulture species from central Spain. Differences were statistically significant in the griffon (Fisher exact tests, *P* = 0.001), cinereous (G-tests, *G* = 18.198, *d.f.* = 1, *P*<0.0001) and Egyptian (G-tests, *G* = 11.778, *d.f.* = 1, *P* = 0.001) vultures. Sample size is shown above bars.

Monitoring until fledging detected the deaths of several nestling griffon (1 of 50) and cinereous (4 of 49) vultures. Necropsy and post-mortem investigations revealed that nestling cinereous vultures that died in the nests were severely infected by the same pathogens found during sampling (*n* = 4, prevalence of *Candida albicans* = 100%, *Aspergillus fumigatus* 25%, *Salmonella* sp. 50%, total prevalence = 100%). Five more cinereous vultures that had been sampled in their nests were found dead or ill in the countryside at various times after fledging. Dead and sick fledgling cinereous vultures were examined in wildlife rehabilitation centres and the latter were treated for severe infections by *C. albicans* (prevalence = 100%, *n* = 5), from which they probably would have died without human intervention. All the sick or dead griffon (*n* = 1) and cinereous (4 nestlings and 5 fledglings) vultures showed antibiotics in plasma when they were sampled in their nests. This suggests an association between fatal disease and the presence of antibiotics in cinereous vultures (Fig. 2).

**Figure 2:** Relationships between the presence of antibiotics in plasma of nestling cinereous vultures and their subsequent survival (Fisher exact test, *P* = 0.006). Sample size is shown above bars.

In addition, nine other cinereous vultures from the same colony that had not been sampled for blood in their nests had one to three antibiotics in their plasma when presented to the rehabilitation centre (see above) and showed severe disease due to the tested pathogens (prevalence of *C. albicans* 78%, *A. fumigatus* 22%, total prevalence = 100%).

### Post-mortem findings and histopathology

External examination of nine cinereous vulture carcasses revealed cachexia, dehydration and poor development. Cultures in standard fungal media showed all had multiple oral, pharyngeal and oesophageal necrotic mucosal plaques caused by *C. albicans*, as well as upper digestive tract congestion and swelling. Macroscopically the liver was enlarged, congested and friable, and the kidney was enlarged and pale pink with white, “chalky” deposits.

Histopathological examinations revealed lesions in the liver and kidney and severely depleted lymphoid organs. Seven out of nine individuals (78%) had vacuolar degeneration of the liver parenchyma and deformed trabeculae. Five individuals (56%) had hyperplasia and fibrosis of the bile ducts with mononuclear infiltrates.

All nine individuals had glomerulonephritis and glomerulonephrosis, mucosal hyperplasia and mild heterophilic inflammation in their renal pelvises and proximal ureters. Six individuals (67%) had mononuclear infiltrates in their renal tissues and a clearly visible tubular epithelium with areas of degeneration and necrosis. Large white aggregates obscured the renal architecture (glomeruli, distal convoluted tubules and collecting tubules) in all individuals but inflammation was minimal. There were extensive diffuse white precipitates on the surface and within the renal parenchyma, consistent with visceral gout, in seven individuals (78%).

## Discussion

Antibiotic bacterial resistance in wildlife has been highlighted as evidence of the impact of increasing human intrusions on wildlife habitats [6], [14]. In this study we demonstrated residues of four different antibiotics in three species of wild birds. To our knowledge, this is the first report of circulating antibiotic residues in wildlife. This striking finding furthers our knowledge about the impact of human activities on environmental health through the potential detrimental effects of circulating antibiotics on wildlife, including the selection and dissemination of antibiotic resistant bacteria.

Avian scavengers ingested antibiotics present in the livestock carrion upon which they feed. Veterinary antibiotics are used in large, although regionally variable quantities throughout the world [15], [16]. Therefore, the potential impact of antibiotic residues on scavenging wildlife may be widespread but the severity is likely to vary with the features of livestock operations and practices of eliminating livestock residues in different regions [8], [9]. The use of different antibiotics to treat livestock in the study area and their variable kinetics may explain their varying presence in each vulture species. Both amoxicillin and oxytetracycline were displaced by quinolones as the drugs of choice alone or with other antibiotics [17], [18], which may explain their high presence and concentrations. The detection of quinolones with other antibiotics in several samples may indicate their combined use and the metabolic transformation of enrofloxacin to ciprofloxacin in livestock and vultures. Differing prevalences and concentrations of antibiotics in the three vulture species may reflect their different feeding habits and physiology, especially the pH of the digestive tract. Griffon vultures evolved as social consumers of entire corpses of large herbivores [19], which has been argued to be associated with the evolution of a very acidic gastric pH (between 1 and 2) to minimise infection by pathogens from rotten meat [20]. Cinereous and Egyptian vultures evolved as scavengers and opportunistic predators of small vertebrates, and preferentially feed upon small fragments of livestock carcasses, especially tendons, skin and viscera [19] which tend to concentrate these antibiotics [21]. The differing ecological and evolutionary strategies for carrion exploitation may explain the different impacts of antibiotics on the health of griffon *vs.* cinereous and Egyptian vultures. Griffon vultures would degrade more antibiotics and pathogens with such a highly acidic gastric pH. This may explain the lower prevalence of antibiotics and pathogens despite the species' greater dependence on livestock carrion. The less acidic gastric pH of cinereous and Egyptian vultures may make them more susceptible to the direct effects of ingested antibiotics despite their higher dependence on wild prey [19].

The mean quinolone concentrations found in vulture plasma may equal that expected in birds treated with a therapeutic dose 24–48 h before testing [22]–[24]. Such high antibiotic concentrations in vultures may indicate an intensive use of these drugs in farming operations in the study area. Antibiotic ingestion is likely to vary with the frequency of use of carrion from different livestock species or wild prey by parental vultures and the concentrations of antibiotics in different livestock carcasses. Nestling vultures may be fed every several days and antibiotics may be metabolised and excreted by birds over a similar time period. This may explain the lack of antibiotics in several nestlings despite the consumption of livestock carrion by all individuals.

The most striking result of this study was the clear association between antibiotic residues, especially quinolones, and disease in the three vulture species. Potential negative health effects of direct antibiotic ingestion with livestock meat include immunosuppression, toxicity, allergy and bacterial flora alteration which may temporarily reduce host resistance to pathogens [1], [23], [24]. The presumably discontinuous ingestion of different antibiotics at different concentrations may lead to sideeffects similar to health problems resulting from the misuse of antibiotics in humans and domestic animals [1], [22]–[24]. For instance, severe infections with *C. albicans* or *A. fumigatus* may be important causes of morbidity and mortality among individuals ingesting antibiotics which enhance the invasiveness of these and other pathogens by altering the normal flora and by depressing the host defences [1], [24].

The impact of antibiotics on the health of cinereous vultures was clearly illustrated by post-mortem findings and histopathology of both liver and kidney samples. All liver samples from dead cinereous vultures contained both enrofloxacin and ciprofloxacin. Although there is no detailed information about the pathology caused by antibiotics in birds, lesions and tissue damage in the liver and kidney are consistent with the expected direct toxic effects of antibiotics in these organs in humans [25]–[28], especially because in birds they concentrate these drugs [21]–[22]. In addition, the severe depletion of lymphoid organs may indicate immunosuppression directly by antibiotics [23]–[24] which may be related to the acquisition and proliferation of the recorded pathogens, even causing severe lesions as in the case of *C. albicans*.

The detrimental effects of ingested antibiotics including the acquisition of pathogens may decrease the health of vultures with a lethal potential, especially in nestlings and fledglings as reported in cinereous vultures. This effect may be associated with the recent steady decline of vulture populations in the study area, especially of cinereous and Egyptian vultures [12], [29]. Therefore, the ingestion of antibiotics in livestock carrion represents a major concern for the conservation of these species. Antibiotic residues in meat in livestock dumps used by scavengers should be regulated to avoid damaging the health and conservation of vultures. The intensive use of antibiotics worldwide and their presence in wild birds have global implications for conservation and in generating and spreading resistant pathogens throughout the environment.

## Materials and Methods

### Fieldwork

We sampled nestlings of the three vulture species breeding in central Spain (primarily in Segovia Province) from 2003 to 2005. In this area a large population of avian scavengers depends on livestock farming providing carrion [8], [9], [29], especially in Segovia province, which has the highest concentration and number of fattening pigs in Spain.

Vulture nests were accessed by climbing and nestlings were sampled at 60–80 days of age, depending on the species. A sample of blood (5 ml) was taken from the brachial vein, centrifuged and the plasma frozen until analysed. Bacterial microflora were sampled from the cloaca, choana and nares of nestlings with sterile microbiological swabs and Amies transport medium. Samples were transported in a chilled container to the laboratory within 12 h after collection and were processed within one to two hours of arrival.

Nestlings were monitored with telescopes until fledging to assess their survival in the nest. Several of these nestlings were found dead in the countryside one or two months after fledging or they were found ill and admitted to wildlife rehabilitation centres where their health status was assessed, including determining the presence of bacterial and fungal pathogens and of antibiotics in plasma. In addition, eight fledglings and one adult cinereous vulture from the same colony as the sampled nestlings (as demonstrated by their rings), which had not been sampled for blood in their nests were found ill in the countryside and admitted to a rehabilitation centre in Madrid between 2002 and 2005. Similar samples were also taken from these individuals.

### Necropsy and histopathological examination

Nine dead nestling cinereous vultures found in or around nests were necropsied and samples of lesions and selected tissues (liver, kidney, lungs, thymus, spleen, gonads, bursa of Fabricius and heart) were collected and fixed in 10% neutral buffered formalin for histopathological examination. Liver samples from each were also taken and frozen at −20°C for the determination of quinolone residues.

### Antibiotic residues in livestock carrion

The Four Plate Test of bacterial growth inhibition to detect antibiotic residues was used on swine tissues (liver, muscle, kidney, oral mucosa, rectum) from seven carcasses found in several livestock refuse dumps where vultures usually forage. This test is extremely sensitive to antibiotics and therefore is routinely performed in slaughterhouses to quickly confirm the presence of antibiotics in food animals [30]. Samples were collected with sterile microbiological swabs, transported in a chilled container to the laboratory within 12 h after collection and processed within one to two hours of arrival. The test was performed in plates with *Bacillus subtilis* spore suspension and *Kocuria rhizophila* bacterial suspension (Merck). Media used to test for residues included test agar pH 6.0 (Merck, dehydrated medium 10663), test agar pH 7.2 with the addition of trimetoprim (Merck, dehydrated medium 15787), and test agar pH 8.0 (Merck, dehydrated medium 10664). Media were prepared according to the manufacturer's instructions. After cooling the agar to 45–55°C, cell and spore suspensions were added to the appropriate media. Sterile standard Petri dishes were filled with 8 ml of the inoculated media and stored at 2–5°C for a maximum of five days.

### Antibiotic residue determination

The presence and concentrations of antibiotic residues in plasma were determined using HPLC techniques and standard protocols [31]–[33]. Briefly, for enrofloxacin and ciprofloxacin, plasma samples (300 µl) were added with an internal standard (75 µl ofloxacin), mixed and shaken with chloroform (4.5 ml). After centrifugation the organic phase was collected and dried under nitrogen. The extracted sampled was injected directly into the HPLC (UV) apparatus (Spectra System AS1000 Autosampler, Thermo Separation Products, Florida USA). These antibiotics were detected using ultraviolet spectrophotometry at 279 nm. The limits of quantification of both molecules were 0.005 µg/ml and the method was linear up to 30 mg/L. The mean percentage recoveries of enrofloxacin and ciprofloxacin were 93% and 90%, respectively. The inter- and intra-assay reproducibility was below 4%.

Liver samples used to determine quinolone residues were homogenised in methanol and centrifuged for pellet debris. Three millilitres of the supernatant were then passed through a solid phase extraction cartridge. Elution was concentrated to a volume of 1 ml. Quinolone concentrations were determined using the same methodology as for plasma samples. The recovery, limit of detection, accuracy and precision of this method were evaluated at concentrations from 0.025 to 250 µg/g. The method was validated and shown to be linear in the range of 0.01–50 µg/g. Spike recoveries for liver prepared at 4 spiking levels ranged from 81% to 98%. The coefficient of variation for recovery as a measure of relative variability was between 3% and 8% and the relative standard deviation was <11%. The limits of quantification were 0.1 µg/g for enrofloxacin and 0.25 µg/g for ciprofloxacin.

For amoxicillin determination, 50 µl of plasma were mixed with 50 µl of perchloric acid using a vortex mixer and then centrifuged to precipitate plasma proteins. The clear supernatant was then injected into the HPLC. Amoxicillin was eluted with a mobile phase consisting of 6% methanol plus phosphate buffer with pH adjusted to 3.2. The concentration of amoxicillin was scanned at a wavelength of 227 nm, and the injection volume was 20 µl. The limit of quantification was 0.05 µg/ml in plasma. The absolute recovery of amoxicillin was 93%. The intra- and inter-assay coefficients of variation were 2% and 3%, respectively.

To determine oxytetracycline concentrations, 9.5g of Mueller-Hinton medium were dissolved in 250 ml of distilled water and autoclaved at 121°C for at least 15 minutes. The solution was cooled to 50°C in a water bath and 0.4 ml of spore solution (1 ml of *B. cereus* spores in 50 ml sterile saline) was added. After the agar solidified 90 µl wells were cut into the bioassay plates. Plasma samples were deproteinised by adding 20 µl of a 30% trichloroacetic acid solution to 40 µl of plasma. The mixture was gently vortexed and centrifuged and the supernatant was assayed. Ninety microlitres of standards, controls and samples were pipetted into duplicate wells in the bioassay plates. Assay plates were incubated at room temperature overnight and the zones of inhibition were measured in micrometres using electronic digital callipers. The plasma concentration was calculated from a standard curve. The limit of quantification was 0.05 µl/ml. Quality control samples were spiked at 0.2, 0.8 and 8 ppm and assayed on each plate.

### Pathogen determination

We determined the presence of two bacterial (*Mycobacterium avium, Salmonella* sp.) and two fungal (*C. albicans*, *A. fumigatus*) species due to their known severe pathogenicities in birds [34] and their potential to proliferate following the ingestion of antibiotics through the alteration of normal flora [1], [9], [34]. To culture *M. avium*, cloacal and tracheal samples taken with sterile swabs were plated on Lowenstine-Jenssen media and incubated for three months. Ziehl-Nielsen and auramine rhodamine acid-fast stains and PCR techniques were used to identify any *Mycobacterium* grown [35], [36]. The presence of a mycobacterium was confirmed if both cultures and molecular techniques were positive. *C. albicans* and *A. fumigatus* were cultured in standard fungical media (Agar Sabouraud) at 37°C for 48 h. Only clinical *C. albicans* was considered, which was determined by the presence of lesions in the oral cavity. For *Salmonella*, samples were cultured and identified to serotype following standard methods described in detail elsewhere [9].
